# Platelet-Rich Plasma for Sport-Active Patients with Knee Osteoarthritis: Limited Return to Sport

**DOI:** 10.1155/2020/8243865

**Published:** 2020-01-31

**Authors:** Sante Alessandro Altamura, Alessandro Di Martino, Luca Andriolo, Angelo Boffa, Stefano Zaffagnini, Annarita Cenacchi, Maria Stella Zagarella, Giuseppe Filardo

**Affiliations:** ^1^Clinica Ortopedica e Traumatologica II IRCCS Istituto Ortopedico Rizzoli, Bologna, Italy; ^2^Servizio Trasfusionale Unico Metropolitano, Bologna, Italy; ^3^Applied and Translational Research (ATR) Center IRCCS Istituto Ortopedico Rizzoli, Bologna, Italy

## Abstract

**Objective:**

To evaluate a cohort of sport-active patients suffering from cartilage degeneration and OA, in terms of clinical outcome and return to sport (RTS) after platelet-rich plasma (PRP) injective treatment.

**Design:**

This study included forty-seven sport-active patients ≤50 years old with unilateral symptomatic knee cartilage degeneration or OA. Patients received 3 PRP injections and were prospectively evaluated at baseline and then at 2, 6, 12, and 24 months follow-up by IKDC subjective EQ-VAS, and Tegner scores. Furthermore, patients were asked about their RTS, in terms of return to any sport level or to their activity level before symptoms onset.

**Results:**

IKDC subjective score improved significantly at all follow-ups, changing from 59.2 ± 13.6 to 70.6 ± 13 at 12 months and to 76.7 ± 12.5 at 24 months (*p* < 0.0005). A similar outcome was observed with the EQ-VAS score. Tegner score improved from 3.6 ± 1.4 to 4.8 ± 0.9 at 24 months (*p* < 0.0005). A similar outcome was observed with the EQ-VAS score. Tegner score improved from 3.6 ± 1.4 to 4.8 ± 0.9 at 24 months (*p* < 0.0005). A similar outcome was observed with the EQ-VAS score. Tegner score improved from 3.6 ± 1.4 to 4.8 ± 0.9 at 24 months (*p* < 0.0005). A similar outcome was observed with the EQ-VAS score. Tegner score improved from 3.6 ± 1.4 to 4.8 ± 0.9 at 24 months (

**Conclusions:**

Sport-active patients affected by knee OA can benefit from PRP injections, with pain and function improvement over time. However, results are less satisfactory in terms of RTS since only half can achieve the same sport level as before the onset of symptoms. Patients undergoing PRP treatment should be made aware of their low chances to go back to high-impact sport activities.

## 1. Introduction

Osteoarthritis (OA) is a common orthopaedic condition characterized by joint pain and decreased function, generally affecting patients over 50 years old: about 25% of ageing people experience pain and other OA-related symptoms, which may be severe and negatively affect their quality of life and productivity, with a high social and economic impact [1–5]. Moreover, an increasing incidence of cartilage degeneration and OA, often related to sport activity, has also been observed in younger patients [6]. In fact, chondral lesions and OA are among the most common causes of knee pain and performance deterioration in athletes, and previous studies have shown a higher incidence of knee OA in athletes compared to the general population [3, 6]. The reason can be found in the continuous cartilage solicitation during physical activity, leading to its premature degeneration with subsequent exposure of subchondral bone that is particularly rich in nociceptive receptors. Furthermore, cartilage damage may cause the release of catabolic and proinflammatory factors generating a vicious circle of painful joint degeneration [7], finally forcing athletes to quit sport.

Total knee arthroplasty represents a common end stage solution for older patients affected by OA, but it does not represent a suitable option in younger patients, due to their high expectations and functional demands. In fact, whereas knee arthroplasty can offer a satisfying functional recovery in older patients, younger patients achieve worse results, with significantly more functional limitations and risks related to the high incidence of failure and the need for subsequent revision arthroplasty [8]. Recently, a database study on 54.000 knee arthroplasties showed that joint replacement in patients under 55 years old increased the lifetime risk for revision up to 35%. This is questioning the impact of the increasing trend of more knee replacements in the younger patient's population [9]. Unfortunately, although alternative surgical procedures relying on scaffolds, tissue engineering, and cell transplantation have shown promising results in young patients with traumatic lesions, they provide less satisfying results and a low rate of return to sport in sport-active patients affected by cartilage degenerative lesions and OA [10, 11].

Intra-articular injective treatments emerged as an alternative minimally invasive option to provide a clinical benefit and delay more sacrificing procedures while avoiding the impact and risks of surgical treatments in these active patients. In the past few years, platelet-rich plasma (PRP) has been proposed for the treatment of knee OA and its use is now supported by increasing evidence [12–17]. Its rational lays on its anabolic and anti-inflammatory properties due to growth factors and cytokines released by platelets [18–21]. Preclinical evidence showed that PRP might promote a favorable environment for joint tissue healing [22]. Nevertheless, although recent reviews and meta-analysis showed good results using PRP for the treatment of OA [16, 22–24], the literature is still very sparse on the use of PRP for the treatment of active patients, and more evidence is needed to document potentials and limitations in this population, both in terms of clinical improvement and return to sport.

Thus, the aim of this study was to evaluate a cohort of sport-active patients suffering from cartilage degeneration and OA, in terms of clinical outcome and return to previous sport activities after PRP injective treatment.

## 2. Materials and Methods

### 2.1. Patients Selection

This study was approved by the Hospital Ethics Committee and the Internal Review Board (blinded) and written informed consent was obtained from all participating patients. Patients were enrolled according to the following inclusion criteria: (1) unilateral symptomatic knee with history of chronic pain (at least 4 months) or swelling, (2) imaging findings of cartilage degeneration (Kellgren–Lawrence score of 0 but with chondropathy detected by magnetic resonance imaging) or OA (Kellgren–Lawrence score of 1-3) (3) playing a sport at any level, (4) ≤50 years old. The exclusion criteria were age greater than 50 years, Kellgren–Lawrence score more than 3, major axial deviation (varus 5°, valgus 5°), focal chondral or osteochondral lesion, presence of any concomitant knee lesion causing pain or swelling (i.e., meniscal or ligamentous injury), inflammatory arthropathy, hematological diseases, severe cardiovascular diseases, infections, immunodepression, treatment with anticoagulants or antiaggregants, use of nonsteroidal anti-inflammatory drugs in the 5 days before blood harvesting, hemoglobin lower than 11 g/dL, and platelet count lower than 150,000/mm^3^.

Forty-nine patients were included; two were lost at follow-up while 47 were evaluated over time, with a mean age at treatment of 41.1 ± 7.1 years and a mean BMI of 25.0 ± 3.0; 15 patients had previously undergone knee surgery and 12 had received injective treatment with hyaluronic acid or corticosteroids.

### 2.2. Patients Treatment and Evaluation

This study was performed at the outpatient department of a highly specialized orthopedics referral center. A single 150 mL unit of peripheral venous blood was harvested from each patient at our Hospital Transfusion Medicine Service. Samples were centrifuged twice: first at 1480 rpm for 6 minutes to separate erythrocytes and then at 3400 rpm for 15 minutes to concentrate platelets, which provided 20 mL of PRP divided into 4 small 5 mL units. One unit was sent to the laboratory for quality tests, and 3 units were stored at −30°C to be used later for treatment, after being thawed in a dry thermostat at 37°C for 30 minutes. Before the injection, PRP was activated by adding 10% calcium chloride. This preparation method was previously shown to reach a number of platelets per milliliter 4.6 ± 1.4 times higher than its baseline blood values and a mean concentration of leukocytes of 1.1 ± 0.5 times compared with normal blood values [25].

Patients received 3 weekly intra-articular injections of PRP. After the injection, they were sent home with indications to use ice or other cold therapy on the affected area to relieve pain and to avoid high-impact activities on the treated leg. After the injections, mild activities were allowed, and, subsequently, a gradual return to normal sport or recreational activities was allowed as tolerated. Patients were prospectively evaluated at baseline and then at 2, 6, 12, and 24 months after their last injection; this evaluation included International Knee Documentation Committee (IKDC) subjective score, EuroQol visual analog scale (EQ-VAS), and Tegner score. Furthermore, patients were asked about their return to sport during the follow-up period, both in terms of return to any sport level or to their activity level before symptoms onset.

### 2.3. Statistical Analysis

All continuous data were expressed in terms of mean and standard deviation of the mean, and the categorical data were expressed as frequency and percentages. The Saphiro–Wilk test was performed to test the normality of continuous variables. The Levene test was performed to assess the homogeneity of variances. The Repeated Measures General Linear Model (GLM) with Sidak test for multiple comparisons was performed to assess the differences at different follow-up times in the IKDC subjective score and the Tegner score. The Friedman nonparametric test, followed by the Wilcoxon post hoc pairwise comparison corrected by Bonferroni method for multiple comparisons, was used for the differences at different follow-up times in the EQ-VAS score and the objective IKDC. The ANOVA test was performed to assess the between-groups differences of continuous, normally distributed and homoscedastic data; the Mann–Whitney test was used otherwise. The ANOVA test followed by the Scheffè post hoc pairwise comparison was also used to assess the among groups differences of continuous, normally distributed and homoscedastic data, the Kruskal–Wallis test followed by the Mann–Whitney test with the Bonferroni correction for multiple comparison was used otherwise. The Spearman Rank Correlation was used to assess the correlation between age or BMI and the observed scores.

For all tests *p* < 0.05 was considered significant.

All statistical analysis was performed using SPSS v.19.0 (IBM Corp., Armonk, NY, USA).

## 3. Results

No major adverse events were reported after treatment, and a statistically significant improvement in all scores was observed.

In particular, the IKDC subjective score improved significantly at all follow-up times compared to the basal evaluation, changing from 59.2 ± 13.6 to 68.0 ± 13.9 at 2 months, 69.9 ± 13.8 at 6 months, 70.6 ± 13 at 12 months, and reaching a maximum of 76.7 ± 12.5 at 24 months (all *p* < 0.0005). Furthermore, the IKDC score at the last follow-up (24 months) was significantly higher than in all other follow-ups (*p*=0.032 vs. 12 months) (Figure 1).

The EQ-VAS score also showed a statistically significant improvement from 73.6 ± 11.9 at basal evaluation to 80.6 ± 11.6 at 2 months (*p*=0.004), 82.2 ± 9.1 at 6 months (*p* < 0.0005 vs. basal), and 81.0 ± 10.4 at 12 months (*p*=0.001 vs. basal), with a further improvement at 24 months follow-up (85.5 ± 8.6, *p* < 0.0005 vs. basal, *p*=0.05 vs. 12 months follow-up) (Figure 2).

The activity level, evaluated by Tegner score, showed a statistically significant improvement from pretreatment level (3.6 ± 1.4) to 2 months follow-up (4.4 ± 1.4, *p*=0.002), with scores remaining stable over time and reaching 4.8 ± 0.9 at the 24 months follow-up (*p* < 0.0005 vs. basal). The activity level after treatment did not reach the level before the onset of symptoms (6.6 ± 1.4, *p* < 0.0005) (Figure 3). Regarding RTS, 36 patients (76.6%) returned to some kind of sport activity, 23 patients (48.9%) were able to return to the same presymptoms activity level.

Further analysis was performed to investigate parameters influencing the clinical outcome at the final follow-up. The Spearman correlation showed that Age and BMI did not significantly influence the score obtained. The Mann–Whitney test showed that previous surgery and previous intra-articular injections did not significantly influence the score obtained. With regard to RTS, rates were not affected by BMI, previous surgery, or previous intra-articular injections. Conversely, a lower presymptoms Tegner score was associated with a higher rate of RTS, both at any level (*p*=0.024) and at the same presymptoms level (*p* < 0.0005).

## 4. Discussion

The main finding of this study was that PRP injective treatment provided a significant clinical improvement in a cohort of sport-active patients affected by OA, allowing the majority of them to return to some sport activity. However, only half of them were able to return to the same level of sport activity as before the onset of symptoms.

The sport-active population affected by knee OA represents a challenge for clinicians, due to the presence of impaired knees in relatively young patients who still have high expectations and functional requirements. In this light, the use of platelet derived growth factors has been proposed as a promising treatment, providing anti-inflammatory and anabolic effects, while avoiding the impact and risks of surgical strategies to address OA [6]. The use of PRP to treat knee OA is being supported by increasing evidence. Its safety and efficacy were proved in randomized controlled trials versus placebo, proving the effects of PRP, with pain reduction and improvement in function and clinical scores at short-term follow-up [12, 14, 15, 26–29]. However, in terms of efficacy in addressing OA joints, the evidence about any possible superiority of PRP versus hyaluronic acid (HA) is more controversial. PRP was first shown to be more effective in reducing pain than HA injections at six months follow-up in a randomized controlled trial by Sánchez et al. [30] in 2012. The same results were confirmed in the same year by Cerza et al. [31] in a large randomized controlled trial on 120 patients. In the following years, a recent review [24] and several other trials confirmed these findings [12, 14, 17, 32] showing, besides no increased risk of adverse events, a significant improvement in short-term exceeding what is considered a minimum clinically important difference.

However, the literature currently lacks evidence on the potential of PRP for the treatment of knee OA in sport-active patients. This is particularly important, as functional sport requirements might be difficult to reach, and positive findings in the overall population cannot be directly translated to sport-active patients. Investigating this aspect is of major importance also in consideration of the controversial results documented for PRP for other sport-related pathologies, that is, tendon and muscle injuries [33, 34]. In the literature, only one research specifically focused on this topic. In a randomized controlled trial, Papalia et al. [35] compared PRP and HA outcomes in a cohort of 47 end career professional soccer players, 23 receiving PRP and 24 HA. They observed a significant improvement in clinical scores and reduction of pain in both groups, with no statistical difference at 12 months follow-up. Although PRP showed some efficacy even in this challenging population, results were limited. Moreover, results were reported only at short-term follow-up, without documenting treatment effect duration. This is an important aspect, as the benefit of PRP is controversial at the longer term, as shown by a recently published randomized double-blind trial questioning the overall benefit of this approach in terms of improvement entity and duration [36]. Finally, this trial did not address one of the major outcomes for these demanding patients, as it did not properly assess sport and activity level and, in particular, return to preinjury sport level.

Return to sport actually represents one of the most important outcomes for this type of patients. In the present study, 47 sport-active patients were treated with 3 injections of PRP and evaluated for up to 24 months of follow-up, not only looking at clinical scores but also addressing specific sport-related questions. In this population, a significant improvement in all scores was reported without significant adverse events related to treatment, confirming the evidence present in the literature that suggests that PRP is safe and effective to treat knee OA [16, 22, 23]. Moreover, results further improved after 12 months: IKDC and EQ-VAS continued to improve over time, with a significant difference between 12 months follow-up and 24 months follow-up. This is an important aspect, previously underinvestigated in the literature, which could be explained with the effects induced by PRP at the joint level. The reduction of inflammation as well as anabolic stimulation might favor the normalization of joint homeostasis: this can allow active patients to go back to sport activity, which in turn could further help maintaining joint function and therefore clinical improvement, as supported by the positive effects of exercise for the management of OA [37].

Sport-active patients affected by knee OA can benefit from PRP injections, with pain reduction and function improvement over time. However, this benefit does not directly translate into a successful sport-related outcome, which represents the most important goal for active patients aiming at returning to sport activity. Despite experiencing some benefits, only 3 out of 4 patients returned to some kind of sport activity, and actually only half of them were able to return to the same activity level. These aspects can be explained considering that sportive patients with OA are likely to reduce their activity level because of OA-related symptoms, and this is generally worsening over time, as a consequence of this suboptimal training practice. On the other hand, it is also true that patients performing contact or pivoting sports subject their joints to higher stress, which could maximize this negative influence of aging. The challenge to improve joint status at a level necessary for sport activity via PRP injection is further supported by the analysis of factors influencing RTS. In fact, the previous activity level was found to be the most important aspect related to the chance to RTS at 24 months of follow-up. In particular, patients with a lower presymptoms Tegner score had more chances to RTS, both at any level and at the same presymptoms level. This means that the more demanding the activity on the joint is, the more difficult it is to provide a sufficient benefit by PRP injections. Thus, when PRP treatment is successful patients might go back to some sport, but often they adapt their activity level, as suggested by the low average Tegner score reached, which mainly corresponds to low impact or no-contact sport activities, even if it is probably not the best evaluation score to thoroughly investigate this aspect.

The present study has some limitations: no comparison with a control group was performed. Considering the limited results documented, further studies should explore PRP injections in the sport-active population also in light of the results provided by other alternative options. Moreover, no imaging evaluation was performed to document the effects of PRP at the tissue level, since the main purpose of this study was to investigate the sport activity level. Finally, the series was large enough to demonstrate an overall significant improvement and the potential in terms of RTS, but it might be insufficient (power <0.4) to find possible differences related to other aspects, such as results in different subpopulations according to age, sex, activity level, and so forth.

Despite the aforementioned limitations, the results of this study are of clinical relevance as they document, in the largest cohort on this topic, and specifically focusing on RTS after up to 24 months, the potential of PRP in the sport-active population. These patients should have the right expectations, as they might experience a clinical improvement insufficient to recover their full function.

## 5. Conclusions

Sport-active patients affected by knee OA can benefit from PRP injections, with good results over time both in terms of pain and function improvement. However, results are less satisfactory in terms of RTS since only half of the patients can achieve the same sport level as before the onset of symptoms. RTS is challenging and patients undergoing PRP treatment should be aware of the low chances to go back to high-impact sport activities.

## Figures and Tables

**Figure 1:** IKDC subjective score at basal level, at 2, 6, 12, and 24 months follow-up.

**Figure 2:** EQ-VAS score at basal level, at 2, 6, 12, and 24 months follow-up.

**Figure 3:** Tegner score at presymptoms and basal pretreatment level, at 2, 6, 12, and 24 months follow-up.

## Data Availability

The data generated during the current study are available from the corresponding author upon reasonable request.
